The article "Numerical Assessment of a Safety System to Minimize Injuries during a Cyclist Run-Over" was published in 2021. Journal: Appl Bionics Biomech.

# Numerical Assessment of a Safety System to Minimize Injuries during a Cyclist Run-Over

**DOI:** 10.1155/2021/9922210

**Published:** 2021-08-26

**Authors:** E. H. López-García, M. F. Carbajal-Romero, J. A. Flores-Campos, C. R. Torres-SanMiguel

**Affiliations:** ^1^Instituto Politécnico Nacional, Escuela Superior de Ingeniería Mecánica y Eléctrica Sección de Estudios de Posgrado e Investigación, Azcapotzalco, 02519 CDMX, Mexico; ^2^Instituto Politécnico Nacional, Unidad Profesional Interdisciplinaria en Ingeniería y Tecnologías Avanzadas, 07340 CDMX, Mexico; ^3^Instituto Politécnico Nacional, Escuela Superior de Ingeniería Mecánica y Eléctrica Sección de Estudios de Posgrado e Investigación, Zacatenco, 07738 CDMX, Mexico

## Abstract

**Background:**

The World Health Organization has reported that 1.35 million people die on the roads every year due to road traffic accidents. This paper focuses on exploring a passive safety system that reduces lesions in the overtaking run-over scenario.

**Methods:**

Head Injury Criterion (HIC) and Combined Thoracic Index (CTI) were evaluated through numerical simulations using LS-Dyna®; in order to compare the computed results, three different speed scenarios were carried out (velocity of running over 40, 50, 60 km/h).

**Results:**

The computed results were divided into groups, A for the run-over test without a passive security system and B for the run-over test with a passive security system. For case A.1, the HIC15 was 3325. For case A.2, the HIC15 was 1510, and for case A.3, the HIC 15 was 1208. For case B.1, the HIC15 2605, for case B.2, the HIC15 was 1282, and for case B.3, the HIC was 730.

**Conclusion:**

The comparative results show that the passive safety system installed on the bicycle has an increased benefit impact on the severity of the injury on vulnerable road users, decreasing the probability of cranioencephalic lesions in all study cases. In addition, the thorax injuries are cut down only in the impact scenario at a speed of 40 km/h.

## 1. Introduction

The World Health Organization (WHO) reported 1.35 million deaths in a year due to road traffic crashes [1]. This problem was the leading cause of death in people between 15 and 29 years in 2012 [2]. A specific group called vulnerable road users (VUR) that include motorcyclist, cyclist, and pedestrians are exposed to a greater danger during their circulation inroads because they do not have any structure that protects them from a road accident and is more susceptible suffer severe or deadly injuries [3]. The cyclist run-over is the smallest group among all road accidents, representing 4% of the victims. Although the numbers of deaths due to the cyclist run-over are a few, it was informed around 52,000 in 2013 [2]. In the United States, 783 cases of cyclist deaths due to motor vehicle crashes were reported in 2017 [4], while in Mexico, the cases of death of cyclists in road accidents totaled 199 in the same year [5]. The cyclist run-over scenarios can be identified according to different characteristics. The Pedestrian and Bicycle Crash Analysis Tool (PBCAT) distinguishes around 79 scenarios that consider different factors such as the vehicle's position before the impact, the direction in which one respects the other, and the impact causes [6]. The scenario reported a greater probability of cyclist death, where the motor vehicle is moving in the same direction as the cyclist and the bicycle is reached in the rear side by the front of the car; this scenario is called the overtaking scenario [7, 8]. Also, in National Highway Traffic Safety Administration (NHTSA) in the database called Fatality Analysis Reporting System (FARS) from 2008 to 2012, the crash scenario that presented the highest death rate of the cyclist in the United States is the overtaking crash scenario [9], repeating this trend in subsequent years until 2017, which is the last update. It is essential to consider the type of motor vehicle studied because this directly affects the severity of the injury that a cyclist can present since its geometric characteristics alter the VUR kinematics. The data issued by the NHTSA show that passenger cars have the second place in deaths caused to cyclists [10–12]. In different industrial designs, existing systems are used to decrease injuries in vulnerable road users, as shown below: the patent [13] presents a bumper used in children's bicycles that has the function of attenuating the frontal collision in front of any surface to protect the bicycle upon impact and reduce the impact force and protect the user. Similarly, the patent [14] presents a pneumatic bumper with an internal chamber that stores air, which is released controlled when the front and rear parts of the bumper cushion impact. Also, the device [15] is designed to be used in motor vehicles. It has two subsystems, an impact mitigation device placed in the front of the vehicle, responsible for absorbing minor impacts that do not exceed the material's yield point, and an internal bumper that deforms plastically and absorbs the impact energy. The patent [16] consists of a U-shaped bumper joined at the motorcycle to protect the vehicle structure from possible shocks. The device [17] is a rigid structure installed on the front or rear of a bicycle to protect the damage by an impact. Finally, the patent [18] shows a bumper placed on the rear wheel of the bicycle, serving as a support for a light source projected towards the ground, marking the minimum safe distance for the circulation of the cyclist to prevent road accidents caused by the lack of vision towards the cyclist.

The research is aimed at proposing a framework used to perform vehicle-bicycle crash simulations to investigate the effects of the rear rubber bumper on cyclist injuries. The novelty is the rear passive safety system rubber bumper and the numerical analysis carried out. The modeling methods used to predict biomechanical responses for run-over simulations are well-established and can help predict biomechanical response in this scenario. A sedan vehicle was chosen for this study due to its high commercial demand and its incidence in cyclists' road accidents. In addition, the head and chest lesions suffered by the cyclist are evaluated since those are the body's main region that causes a person's death in run-over scenarios.

## 2. Materials and Methods

Three cyclists' crash impact simulations were carried out using the finite element method by Ls-Dyna® Software, through a detailed analysis due to the high nonlinearities, the inertial components, and the short duration of the phenomenon. All the simulations are carried out in the overtaking crash scenario, where the car impacts the bicycle's rear wheel while the bicycle and the vehicle are in the same direction [19]. The characteristics for each case of run-over are described in Table 1.

Bicycle and cyclist position was proposed before the vehicle's impact to measure injuries generated under the cyclist's head. The initial position before impact can be seen in Figure 1.

Three meshed models corresponding to the vehicle, bicycle, and cyclist were used, described in detail below. The automobile model consists of a meshed geometry compatible with the Ls-Dyna® software of a Toyota Yaris 2010, developed by George Mason University, contracted by the Federal Highway Administration (FHWA). This model has validations under the various frontal and lateral impact tests and a substantial barrier impact [20]. The anthropomorphic virtual dummy used during the simulations to represent the cyclist run-over scenario corresponds to a male Hybrid III percentile 50th, developed by the Livermore Software Technology Corporation, developing the LS-Dyna® software. The bicycle model was developed in the SolidWorks® Computer-Aided Design (CAD) software to later export the geometry to the LS-Dyna® software, where it proceeded to mesh and configure the corresponding contacts and joints. The bicycle frame was based on the Bicyclist and bike targets specifications manual version 1.1, developed by CATS/4a companies, to provide the necessary specifications of a cyclist objective vehicle detection tests. This research used the size of bicycles for an average man in the Dutch population [21]. The characteristics of the vehicle, dummy, and bicycle model are shown in Table 2.

The bicycle frame and wheel discretization were made with shell elements. The element type used in the model was quadrangular elements with 4 nodes, and we used the mesh algorithm provided by the LS-PrePost® software to create a preliminary mesh, then carried out a manual mesh refinement process to achieve a high mesh quality, especially in areas of interest of the model, where correct discretization is critical for the reliability of the results. To ensure that the quality of the mesh was acceptable, mesh quality checks shown in Table 3 were carried out, where it was observed that the mesh of the bicycle parts had a good quality, especially in critical areas for the results.

The LS-Dyna® software has a large number of material models used for different applications. For this research, to represent the behavior of the metallic parts, bicycle, and the passive safety device, we used the MAT_PIECEWISE_LINEAR_PLASTICITY model. The material selected for the bicycle frame was AISI 4130 steel, a common material for bicycle frames. In order to properly simulate impact behavior, the material's linear and nonlinear mechanical properties are needed to be configured appropriately within LS-PrePost®.  Table 4 shows the parameters necessary to define those mechanical properties.

The bicycle frame was validated through the tests described in Mexican Standards nmx-d-198-2-1985 and nmx-d-198-3-1985, specifically in points 4.3.1 and 4.3.2 corresponding to the mass impact test in frame-scissor assembly and drop of the frame-scissor assembly, respectively, which were performed in LS-Dyna®. The frame drop safety test consists of fixing the frame's rear axle, then a mass (M1) of 70 kg must be fixed on the seat post, and the assembly is dropped on a steel anvil [22]. The conditions necessary for the bicycle frame to be considered safe are as follows:

- The frame must not suffer any visible fracture [22]
- The permanent deformation measured between the initial and final position of the center of the front axle of the wheel must not exceed 60 mm [22]

In the frame impact safety test, a mass (*M*) of 22.5 kg was dropped from a height (*a*) of 180 mm and hit the front part aligned with the centers of the wheels [22]. Therefore, the parameters necessary for the bicycle frame to be considered safe must meet two conditions:

- The frame must not suffer any visible fracture [22]
- The permanent deformation measured between the wheel axles' centers must not exceed 40 mm [22]

Figure 2 shows the diagram for the frame drop safety test and frame impact safety test.

### 2.1. Passive Safety Device

The strain energy density influences the severity of cyclist's injuries. This property quantifies the stored and dissipated energy in a material when it suffers a deformation. This energy is quantified from the different parts of the virtual dummy that represents the cyclist's body. Therefore, the passive safety device seeks to dissipate the most significant deformation energy before the cyclist's body hits the car's surface. The graphic method of material selection is used, also called the Ashby method [24].

The device was based on automotive bumpers systems consisting of a frame, an energy absorber, and a plastic fascia. A passive safety system was designed, consisting of a frame made of ASIS 201 stainless steel and a polyurethane rubber elastic energy absorption system. These materials were chosen due to their high capacity to absorb impact energy. The frame part is responsible for absorbing the most outstanding amount of plastic deformation energy from being run over by a vehicle. In contrast, the polyurethane rubber parts seek to protect minor impacts by absorbing the most significant elastic deformation energy. The assembly of the system is carried out through arrangements of nuts and screws. The system dimensions were established for the bumper's average height, which was used to place the bicycle's passive safety system. Since the average height of a vehicle's bumper is 500 mm [25], the system must be placed within this measurement.  Figure 3 shows how the passive safety system is mounted on a bicycle.

The passive safety device's frame was discretized similarly to the bicycle's frame by using shell elements to optimize computational resources without sacrificing accuracy. Mesh quality check results are shown in Table 2. The material model was again MAT_PIECEWISE_LINEAR_PLASTICITY due to the characteristics already described; the mechanical properties necessary to simulate the correct impact behavior are shown in Table 3. In polymer blocks, the MAT_MOONEY-RIVLIN_RUBBER model specialized in this group of materials was used. The mechanical properties necessary to simulate the behavior of this part of the passive safety device are shown in Table 5.

## 3. Results

The safety framework tests were carried out to bring the following results. First, the front scissors' axis's deformation was measured at the maximum position upon reaching rest (at time *t* = 2000 ms) against the position instants before hitting the rigid wall (at time *t* = 752.0 ms).  Figure 4 shows the stages of the frame drop test and the results, where the maximum deformation was 3 mm, indicating that this value is established by the standard on which the tests are based.

The axis deformation at the front scissors was measured at the maximum position when the impactor is not in contact with the bicycle's frame to measure the permanent deformation in it.  Figure 5 shows the stages of the frame impact test and the results where the permanent deformation (without load) presented in the frontal part of the frame was 16.7 mm, being within the tolerable limits of permanent deformation indicated by the standards on which the simulations are based.

### 3.1. Vehicle-Cyclist Impact Simulations

Bodily, the injuries happen when its resistance exceeds the withstand energy. Thus, for an object to lose speed, its energy of motion must be transferred to another object. This transfer of energy also occurs in the case of an accident in the human body. The kinetic energy dissipated during the cyclist's collision is transformed into the structure deformation, leaving less residual energy to be absorbed for the mechanical properties of the hard and soft tissue. The dispersion of kinetic energy, both in space and in time, is determinant in reducing the severity of injuries and can make the difference between surviving and not. The most severely injured body areas are the head and thorax. In this research, Head Injury Criterion (HIC) and Combined Thoracic Index (CTI) determine the energy generated during the cyclist's collision. These injury rates are calculated according to the following equations.

A suitable measurement to scale the possible cranioencephalic injuries is used the HIC. This criterion reflects the change in acceleration that the passenger's head undergoes moments after the collision. The calculation is performed by selecting the maximum limits of integration of the area under the acceleration curve. NHTSA and AAMA (American Association of Medical Assistants) have established a time interval of 15 milliseconds after the impact. This interval favors the reduction of the HIC calculation error. In addition, this value provides a more rigorous measurement of injury probability.

(1) $$\begin{array}{c} \text{HIC}=\left\{\left(t2-t1\right){\left[\frac{1}{t2-t1}\int_{1}^{2}a\left(t\right)dt\right]}^{2.5}\right\}. \end{array}$$

HIC uses *t*2 and *t*1 as a period of deceleration curve, *a* is the acceleration, and *t* is the total period of the curve. In order to determine a HIC value, it is necessary to obtain the velocity and acceleration of the body at the moment of impact. Therefore, the dummy's dimensional characteristics are crucial to establish a way to generate such kinematic parameters.

Additionally, the Combined Thoracic Index sums the ribs and skin deflection, measured on cadavers using chest bands. However, the chest deflections measured on the dummy represent only the internal chest deflections of the ribs. Thus, the combined thoracic injury criteria, CTI, is defined with the following equation

(2) $$\begin{array}{c} \text{CTI}=\frac{A_{\max}}{A_{\mathrm{int}}}+\frac{D_{\max}}{D_{\mathrm{int}}}, \end{array}$$

where *A*_max_ is the maximum value of 3 ms clip spinal acceleration (As), *D*_max_ is the maximum value of the dummy deflection (*D*), and *A*_int_ and *D*_int_ are the respective intercepts as defined above.

The dummy used has accelerometers in different parts of the body. For example, the accelerometer location in the head is at node 133919, while that of the thorax is node 135705, shown in Figure 6. Those nodes measure the accelerations, and the LSDyna software calculates the HIC and CTI reached during the run-over.

This section shows the results of simulations performed with the characteristics mentioned in Table 6, evaluating the cyclist's head injuries HIC and the CTI index for chest injuries. The simulation results were compared in two cases with the same vehicle's same speed but with and without a passive safety system to observe the injuries differences.

### 3.2. Comparison between Case A.1 and Case B.1

For the case in which the car moves at 60 km/h, Figure 7 shows the kinematic of the cyclist in cases A.1 and B.1, while Table 6 shows the corresponding HIC and CTI values. Finally, Figure 8 shows the required parameters to assess head and thorax injury severity at 60 km/h.

By using the results of the Combined Thoracic Index acceleration of the chest center of gravity as well as chest deflection during a traffic accident, it is possible to know the probability that the cyclist suffers AIS ≥ 3  and AIS ≥ 5 injuries is 99.23% and 43.22%, respectively, for case A.1. For case B.1, the probabilities are 99.58% and 55.77%, respectively.

### 3.3. Comparison between Case A.2 and Case B.2

For the case in which the car moves at 50 km/h, Figure 9 shows the kinematics of cyclists in cases A.2 and B.2, while Table 6 shows the corresponding HIC and CTI values. Finally, Figure 10 shows the required parameters to assess head and thorax injury severity at 50 km/h.

By using the results of the Combined Thoracic Index acceleration of the chest center of gravity as well as chest deflection during a traffic accident, it is possible to know the probability that the cyclist suffers AIS ≥ 3 and AIS ≥ 5 injuries is 94.72% and 13.23%, respectively, for case A.2. For case B.2, the probabilities are 97.37% and 21.54%, respectively.

By obtaining the resulting acceleration graph at the center of gravity of the cyclist's head in both cases, it is possible to know that the HIC15 parameter is 1510 for case A.2, while for case B.2, it is 1282. This difference is because there is less acceleration in the center of gravity of the cyclist's head. After all, the safety device modifies the cyclist's kinematics during a collision, causing that the head hits closer to the center of the vehicle's windshield, as shown in Figure 11(b), which is less rigid than the contour.

### 3.4. Comparison between Case A.3 and Case B.3

For the case in which the car moves at 40 km/h, Figure 12 shows the cyclist's kinematics in cases A.3 and B.3, while Table 6 shows the corresponding HIC and CTI values. Finally, Figure 13 shows the required parameters to assess head and thorax injury severity at 50 km/h.

The HIC and the Abbreviated Injury Scale (AIS) correlation is estimated life-threatening without the passive security system. On the other hand, with the device being installed, the results show that HIC15 turns out to be close to the limit allowed by the Federal Motor Vehicle Safety Standards (FMVSS) [26, 27], and the injuries that the cyclist may have ranged from moderate to minor.

By using the results of the Combined Thoracic Index acceleration of chest center of gravity as well as chest deflection during a traffic accident, it is possible to know the probability that the cyclist suffers AIS ≥ 3 and AIS ≥ 5 injuries is 97.79% and 24.09%, respectively, for case A.3. For case B.3, the probabilities are 80.77% and 4.48%, respectively.

## 4. Discussion

It shows that the kinematics of the cyclist during impact is quite similar to the results obtained in the present work, as shown in Figure 14. In addition, the HIC parameters for cases of 50 km/h and 40 km/h are quite similar when presenting only 9.32% and 6.09% errors, respectively, compared to their tests. Only when the impact is at 60 km/h, the results differ from each other. It can be explained due to the different geometry between the fronts of the vehicles used because the cyclist's head hits a higher area of the windshield at this speed, which has a higher stiffness, which significantly increases HIC. On the other hand, Raslavicius et al. use a multibody solver, while this work uses a finite element model that can make specific differences in body deformations in contact during impact [7]. The results obtained are steady with the severity of the literature's injuries by agreeing that this crash scenario generates severe or fatal injuries [8, 28].

The vehicle model used in this work was validated under the various front and lateral impact tests [20], the dummy model was provided by Livermore Software Technology Corporation, and the bicycle was validated according to the Mexican Standards nmx-d-198-2-1985 and nmx-d-198-3-1985.

A bumper placed at the bicycle's rear mitigates injuries caused by the vehicle's impact on the cyclist and absorbs kinetic energy due to the impact. The system is also useful for changing the body's kinematics. The head hits an area closer to the windscreen center due to the same principle of deformation energy density, being less rigid, reducing the possible severity of craniocerebral injuries. It can be seen that the rate of craniocerebral injury for the scenario with the passive safety device installed on the bicycle is considerably lower, which influences the probability and severity of the injury, going from being incompatible with survival to having a chance of survival. However, with critical and nonreversible injuries, a skull fracture is presented, with a loss of consciousness for more than 24 hours, and intracranial hemorrhage occurs. In the case of the thorax injuries, the two cases' probabilities are similar since it is estimated that there will be a fracture of multiple ribs in both cases. Likewise, there is a 43.22% and 57.77% probability in cases A.1 and B.1, respectively, of complex thoracic injuries with respiratory difficulty, production of massive hemothorax, and cardiac rupture or contusion, which fall into the category of critical injuries with uncertain survival. For the lower limbs, it is essential to mention that only the right limb is referred to in the tables since, due to the setup of the hit-and-run scenarios, and the left lower limb always presents injuries far below those generated in the right limb. Both hit and run cases show similar results, where there is a probability of less than 50% of presenting a nondisplaced fracture of the femur, an injury categorized as moderate on the AIS scale. In comparison, the probability of presenting an exposed fracture of this bone is less than 20% in both cases, although this probability is lower when the bicycle has a passive safety device installed. There are injuries to the cyclist's right tibia; injuries, show an AIS = 2 level injury will undoubtedly occur, indicating a fracture of this bone due to the impact.

The results show the craniocerebral injury rate for the scenario with the passive safety device fitted to the bicycle is again considerably lower, classified on the AIS-4, which is severe, but with probable survival, where cranioencephalic trauma with or without fractures may occur, accompanied by unconsciousness and neurological signs such as posttraumatic amnesia for 3-12 hours. On the other hand, the most likely injuries when the bicycle does not have a passive safety device are categorized at AIS = 5 level, critical injuries where survival is uncertain. In the case of injuries to the thorax, the probabilities between the two cases are again similar, since it is estimated that in both cases, there will be a fracture of multiple ribs, with a probability of practically 100% of presenting an AIS = 3 level injury; likewise, there is a 13.23% and 21.54% probability in cases A.2 and B.3, respectively, with a 13.23% and 21.54% probability of presenting an AIS = 3 level injury, respectively. Moreover, case B.3, respectively, has a 13.23% and 21.54% probability of AIS = 5 thoracic injuries, complex injuries with respiratory difficulty, production of massive hemothorax, and cardiac rupture or contusion, which fall into the category of critical injuries with uncertain survival [29, 30]. For the lower limbs, in this case, there is a considerable difference in the probability of injury to the cyclist's right femur, since in the case where the bicycle does not have the safety device installed, the probability of suffering a nondisplaced fracture is 8.18%.

In comparison, if the device is installed, the probability increases to 28.4%. In presenting an exposed fracture in this bone, the probability remains less than 20% in both cases, although it is higher when the bicycle has a passive safety device installed. The cyclist's right tibia shows an AIS = 2, which indicates the fracture of this bone due to the impact.

The results the tables have shown are again considerably lower, which influences the likelihood and severity of the injury, being categorized on the AIS scale as level 3 injuries that are serious but not life-threatening and are fully reversible, although hospitalization is necessary. On the other hand, the most likely injuries when the bicycle is not fitted with the passive safety device are categorized at AIS level 4, severe, life-threatening injuries, but with probable survival. In the case of injuries to the thorax, the probabilities between the two cases show a more significant variation than in the previous cases, since the probability of suffering an ASI = 3 or greater injury for the case where the bicycle does not have the passive safety device installed is very close to 100% (97.79). In contrast, if the bicycle does have this device installed, the probability decreases to 80.77%. The same pattern is observed in the probability of suffering injuries ASI = 5 or greater, where case A.3 has 24.09%, while case B.1 has 4.48%. For the lower limbs, specifically the cyclist's right femur, the results between both cases are again quite similar, approaching the null probability of injury to the femur, whether AIS = 2 or AIS = 3, with a variation of no more than 2% between the results and a percentage of injury of less than 5%. In the case of cyclist's right tibia, the results again show that an AIS = 2 level injury will occur, which indicates the fracture of this bone injury is a consequence of the impact since the percentage of presenting this injury remains at the same value as the previous cases with a 100% probability of fracture.

For the cranioencephalic injuries generated in the accident, in all cases where the passive safety device was used, the HIC index decreased considerably, reducing the severity of the injuries by one level according to the AIS scale. However, the impact of this is not minor, as it has several implications.

1. In cases where a cyclist is hit at a speed of 60 km/h, the device's use can reduce the likelihood of injury to such a degree that survival is possible, which is not the case where the device is not fitted
2. For the 50 km/h cases, the use of the device can reduce the probability of injury, compared to the results obtained for the run-over cases where the device is not installed, so that the expected injuries correspond to the ASI = 4 level, where survival is likely, as opposed to the AIS = 5 level, where the injuries generated are critical
3. In a collision at a speed of 40 km/h, the injuries generated on the cyclist, when using the passive safety device, are reduced to an AIS = 3 level, where the cyclist's life is not at risk, although the injuries are categorized as severe, whereas without the device, the injuries grow to an AIS = 4 level, where the person is likely to die

The first limitation of this work is the dummy model used. A pedestrian dummy for the collision model was mounted on the bicycle and then used to report the injuries as a vulnerable road user. For this reason, it is important to corroborate the results with a specific case of the study by means of MADYMO® models. Another limitation of this work is the possibility of using THUMS® anthropomorphic dummies to determine the state of stress and deformation of soft tissue and hard tissue. Finally, the most critical limitation is the lack of other experimental dummies to report similar injuries on vulnerable road users. It is then essential to carry out studies with shielding equipment such as helmets and lower limb protectors to corroborate the presented results. An important aspect worth mentioning in this study is the change in the severity of the injury due to the use of bicycle helmets during vehicular accidents. The characteristics and operation of a bicycle helmet do not significantly impact the cyclist's kinematics during the accident until the cyclist's head comes into contact with the car [31, 32].

## 5. Conclusions

The passive safety device significantly reduced the severity of craniocerebral injuries by decreasing the magnitude of the HIC index by 775, 228, and 478 points for impact speeds of 60 km/h, 50 km/h, and 40 km/h, respectively. The passive safety device's use did not significantly reduce the severity of thoracic injuries at high speeds (60 km/h and 50 km/h); however, it did reduce them at low speeds (40 km/h) by obtaining a 19.61% less of the probability of suffering an injury, presenting an AIS ≥ 5 injury when using the device. The forces applied to the cyclist's femur indicated a 28.4% greater variation in the probability of sustaining an AIS ≥ 2 injury when using the passive safety device. In conclusion, the design fulfilled its primary function by reducing the severity of cranioencephalic injuries to one level in the AIS system in all cases, which implies the significant decrease in risk of death by cranioencephalic trauma, especially at low-speed cases in this particular run-over scenario, because this type of injury is the one with the highest risk of mortality for cyclists.

## Figures and Tables

**Figure 1:** Initial position cyclist/automobile.

**Figure 2:** Frame drop safety test and frame impact safety test [23].

**Figure 3:** Passive security system fixed to the bicycle.

**Figure 4:** Front scissors' deformation: (a) initial position of the frame drop test; (b) moment before impact; (c) maximum permanent deformation position; (d) longitudinal displacement of the center of the front scissors' axis for the frame drop test.

**Figure 5:** Frame deformation: (a) frame contact with impactor; (b) moment after contact with impactor (maximum permanent deformation); (c) longitudinal displacement of the center of the front scissors' axis for frame impact safety test.

**Figure 6:** The head and thorax accelerometer location.

**Figure 7:** Impact on a cyclist on the overtaking stage at 60 km/h without a passive safety system (a) and with a passive safety system (b).

**Figure 8:** (a) Acceleration in the head and HIC's gravity center at a speed of 60 km/h. (b) Acceleration of chest gravity center in G's at a speed of 60 km/h. (c) Chest deflection in mm during a traffic accident at a speed of 60 km/h.

**Figure 9:** Cyclist overtaking impact at 50 km/h without a passive safety system (left) and with a passive safety system (right).

**Figure 10:** (a) Acceleration of head gravity center and HIC at a speed of 50 km/h. (b) Acceleration of chest gravity center in G's at a speed of 50 km/h. (c) Chest deflection in mm during the accident at a speed of 50 km/h.

**Figure 11:** Cyclist's head windshield contact at the vehicle. (a) No passive safety device (b) with a passive safety device.

**Figure 12:** Cyclist overtaking impact at 40 km/h without a passive safety system (a) and passive safety system (b).

**Figure 13:** (a) Head acceleration in the center of gravity and HIC at a speed of 40 km/h. (b) Chest acceleration in G's at a speed of 40 km/h. (c) Chest deflection in mm during the accident at a speed of 40 km/h.

**Figure 14:** Cyclist's kinematics during an overtaking crash. (a) MADYMO run-over simulation; (b) FEM simulation.

**Table 1:** Characteristics of run-over tests.

Group A (without passive security system)	Case A.1	
	Automobile speed	Cyclist speed
	60 km/h	0 km/h
	Case A.2	
	Automobile speed	Cyclist speed
	50 km/h	0 km/h
	Case A.3	
	Automobile speed	Cyclist speed
	40 km/h	0 km/h
Group B (with passive security system)	Case B.1	
	Automobile speed	Cyclist speed
	60 km/h	0 km/h
	Case B.2	
	Automobile speed	Cyclist speed
	50 km/h	0 km/h
	Case B.3	
	Automobile speed	Cyclist speed
	40 km/h	0 km/h

**Table 2:** Toyota Yaris 2012 and Hybrid III 50th percentile characteristics [20, 21].

Model characteristics	Yaris 2012	Hybrid 50th	Bicycle
Number of parts	919	115	12
Number nodes	393165	7353	53314
Number of solid elements	15234	2644	—
Number of shell elements	358457	1606	56724
Number of beam elements	4685	3	—
Number of restriction joints	19	48	—

**Table 3:** Mesh quality checks for bicycle and passive security system model.

Variable	Definition	Acceptable value	Percentage of valid elements	Percentage of valid elements
Aspect ratio	The ratio between the largest and smallest dimensions of an element	<10	99.76%	99.86%
Skewness	Angular deviation of the element from an ideal shape	<45°	97.51%	99.95%
Warp angle	The angle between the normal two planes is formed by split the quadrilateral element along the diagonals	<100°	99.36%	99.46%

**Table 4:** Mechanical properties of AISI 4130 and AISI 201 Steel.

Material	Mass density. (Ton/mm^3^)	*E* (MPa)	Poisson's ratio	*σ*_YS_ (MPa)	$\tilde{\sigma_{R}}$ (MPa)	$\tilde{\varepsilon_{f}}$	*n*	*E*_*t*_ (MPa)
AISI 4130	7.850×	205 × 10^3^	0.29	460.00	914.481	0.224	0.1456	2.48
AISI 201	7.810 × 10^−9^	200 × 10^3^	0.27	360.00	1377.5	.03715	0.2099	2.61

*E* = Young′s modulus; *σ*_YS_ = yield stress; $\tilde{\sigma_{R}}=\text{true fracture stress}$; $\tilde{\varepsilon_{f}}=\text{true fracture strain}$; *n* = strain hardening exponent; *E*_*t*_ = tangent modulus.

**Table 5:** Mechanical properties of polyurethane rubber with Mooney-Rivlin formulation.

Mass density (Ton/mm^3^)	Poisson's ratio	*A*	*B*
1.20×	0.27	1.24	0.01

*A* and *B* are the constants of the Mooney-Rivlin constitutive equation for rubber. In the case of polyurethane rubber, the corresponding coefficients are *A* = 1.24 and *B* = 0.01 [26].

**Table 6:** Evaluation of HIC 15 and CTI with and without a passive safety system.

Velocity	Case	HIC15	AIS head	CTI	AIS chest
60 km/h	A.1	3325	AIS ≥ 6	1.933	AIS ≥ 5 = 55.77%
60 km/h	B.1	2605	AIS ≥ 5	2.03	AIS ≥ 5 = 43.22%
50 km/h	A.2	1510	AIS ≥ 5	1.62	AIS ≥ 5 = 21.54%
50 km/h	B.2	1282	AIS ≥ 4	1.73	AIS ≥ 5 = 13.23%
40 km/h	A.3	1208	AIS ≥ 4	1.76	AIS ≥ 5 = 24.09%
40 km/h	B.3	730	AIS ≥ 3	1.39	AIS ≥ 5 = 4.48%

## Data Availability

The data used to support the findings of this study are available from the corresponding author upon request.
